The article "Exosomes from the tumour-adipocyte interplay stimulate beige/brown differentiation and reprogram metabolism in stromal adipocytes to promote tumour progression" was retracted in 2023. Reasons: duplicated images; signs of a paper mill; unreliable results or conclusions.

# Exosomes from the tumour-adipocyte interplay stimulate beige/brown differentiation and reprogram metabolism in stromal adipocytes to promote tumour progression

**DOI:** 10.1186/s13046-019-1210-3

**Published:** 2019-05-28

**Authors:** Qi Wu, Juanjuan Li, Zhiyu Li, Si Sun, Shan Zhu, Lijun Wang, Juan Wu, Jingping Yuan, Yimin Zhang, Shengrong Sun, Changhua Wang

**Affiliations:** 1 Department of Breast and Thyroid Surgery, Renmin Hospital of Wuhan University, 238 Ziyang Road, Wuhan, 430060 Hubei Province People’s Republic of China; 2 Department of Clinical Laboratory, Renmin Hospital of Wuhan University, Wuhan, Hubei People’s Republic of China; 3 Department of Pathology, Renmin Hospital of Wuhan University, Wuhan, Hubei People’s Republic of China; 4 Department of Pathophysiology, Wuhan University School of Basic Medical Sciences, Wuhan, 430060 Hubei Province People’s Republic of China

**Keywords:** Breast cancer, Exosomes, Adipocytes, Tumour progression

## Abstract

**Background:**

Emerging evidence supports the pivotal roles of adipocytes in breast cancer progression. Tumour induced beige/brown adipose tissue differentiation contributes to the hypermetabolic state of the breast cancer. However, the mediators and mechanisms remain unclear.

**Methods:**

Survival probabilities were estimated using the Kaplan–Meier method based on immunohistochemistry results. Biochemical studies were performed to characterize the novel interrelation between breast cancer cells and adipocytes.

**Results:**

We show that tumour-surrounding adipocytes exhibit an altered phenotype in terms of upregulated beige/brown characteristics and increased catabolism associated with an activated state characterized by the release of metabolites, including free fatty acids, pyruvate, lactate and ketone bodies. Likewise, tumour cells cocultivated with mature adipocytes exhibit metabolic adaptation and an aggressive phenotype in vitro and in vivo. Mechanistically, we show that tumour cells induce beige/brown differentiation and remodel metabolism in resident adipocytes by exosomes from the co-culture system that carry high levels of miRNA-144 and miRNA-126. miRNA-144 promotes beige/brown adipocyte characteristics by downregulating the MAP3K8/ERK1/2/PPARγ axis, and exosomal miRNA-126 remodels metabolism by disrupting IRS/Glut-4 signalling, activating the AMPK/autophagy pathway and stabilizing HIF1α expression in imminent adipocytes. In vivo inhibition of miRNA-144 or miRNA-126 decreases adipocyte–induced tumour growth.

**Conclusions:**

These results demonstrate that by inducing beige/brown differentiation and enhancing catabolism in recipient adipocytes, exosomal miRNA-144 and miRNA-126 from the tumour-adipocyte interaction reprogram systemic energy metabolism to facilitate tumour progression.

**Electronic supplementary material:**

The online version of this article (10.1186/s13046-019-1210-3) contains supplementary material, which is available to authorized users.

## Background

Tumour progression is influenced not only by tumour cells but also by surrounding stromal tissues [1]. During breast cancer invasion and metastasis, reciprocal and dynamic communication occurs between tumour cells and the stromal compartments [1]. Specifically, tumours change the normal stroma into an advantageous microenvironment by promoting the wound healing response [2] and are considered metabolic parasites, seizing metabolites such as lactate, pyruvate, fatty acids and ketone bodies from stromal sources [3, 4].

Upon interaction with breast cancer cells, adipocytes, as the main cellular components constituting the breast cancer microenvironment, are transformed into cancer-associated adipocytes (CAAs) and promote tumour progression [5, 6]. Emerging evidence indicates that adipocytes, as endocrine cells, produce abundant inflammatory factors, growth factors, and cytokines, which stimulates receptor tyrosine kinase signalling and epithelial-mesenchymal transition (EMT) programmes [4, 7]. Recently, adipocytes were primarily regarded as tremendous energy storage cells that also provide high-energy metabolites [8]. The metabolic reprogramming of adipocytes may be attributed to their potential tumour promoting ability, and there is speculation that tumours may reprogram adipocyte metabolism to promote disease progression through the dynamic interaction between breast cancer cells and adipocytes.

Exosomes are small (30–100 nm) membrane encapsulated vesicles that are released into the extracellular microenvironment by many cell types, including cancer cells, and represent an important mode of intercellular communication [9]. This cell-to-cell biological communication is mediated through the exchange of the exosome content, which consists of mRNA, ncRNA, transcription factors, proteins, and lipids [10]. Exosomes have been shown to be released by many cancer types, and can be identified through the overexpression of the membrane markers (CD63, CD81 and TSG101, etc.) [10]. In addition, exosomal miRNA profiles parallel those of the originating tumour cells [11]. It is evident that miRNA dysregulation plays a primary role in tumour initiation, progression, and metastasis [12]. Although our previous studies have demonstrated that exosomes derived from tumour cells mediated the metabolic changes in stromal cells and myocytes [13, 14], their potential role in the neoplastic transformation of adipocytes has not been elucidated. Thus, we hypothesize that the underlying mechanism involves the delivery of special miRNAs from breast cells to adipocytes in the breast cancer microenvironment via exosomes, resulting in the conversion of resident adipocytes to CAAs.

Here, we report that adipocytes differentiate towards a beige/brown phenotype and release metabolites, such as lactate, pyruvate, free fatty acids (FFAs) and ketone bodies, upon receipt of cocultivation-derived exosomes to promote tumour proliferation and metastasis. Our data show that specific miRNAs in these exosomes are associated with the pro-tumorigenic process. This work suggests that cocultivation-derived exosomes are novel factors that promote tumour progression by remodelling resident adipocytes towards an activated phenotype through the promotion of beige/brown differentiation and by increasing catabolism in adipocytes.

## Material and methods

### Patients

Human samples were obtained from Renmin Hospital of Wuhan University. Patients did not receive financial compensation. Clinical information was obtained from pathology reports, and the characteristics of the included cases are provided in Additional file 1: Table S1. Patients with at least 5 years of follow-up were included in this study. All methods were performed in accordance with relevant guidelines and local regulations.

### Cell culture and reagents

The human breast cancer cell lines MCF-7 and MDA-MB-231 and HEK 293 T cells were obtained from American Type Culture Collection (ATCC, Shanghai) and cultured in Dulbecco’s modified Eagle’s medium (DMEM) supplemented with 10% exosome-free foetal bovine serum (FBS, Shin Chin Industrial, SCI) and 1% penicillin–streptomycin (HyClone, Logan, UT, USA) in a humidified 37 °C incubator with 5% CO_2_. 3T3-L1 preadipocytes were obtained from ATCC (Shanghai) and cultured in DMEM supplemented with 10% foetal calf serum (FCS, Gibco) and 1% penicillin–streptomycin (HyClone, Logan, UT, USA) in a humidified 37 °C incubator with 5% CO_2_; these cells were differentiated as previously reported [15]. Differentiation was confirmed by Oil Red O staining. Cytochalasin D and insulin were purchased from Sigma.

### Coculture and migration and invasion assays

Mature 3T3-L1 and breast cancer cells were cocultured using Transwell culture plates (0.4-μm pore size; Millipore). Mature 3T3-L1 cells in the bottom chamber of the Transwell system were cultivated in serum-free medium containing 1% bovine serum albumin (Sigma) for 4 h. A total of 3 × 10^5^ MCF7 or MDA-MB-231 cells were cultivated in the top chamber in the presence or absence of mature 3T3-L1 cells in the bottom chamber for the indicated times. Adipocyte conditioned medium (AD-CM) and cancer cell conditioned medium were collected from cells cultivated alone under similar conditions for 3 days and served as controls, while CAA conditioned medium (CA-CM) was collected from adipocytes cultivated with tumour cells for 3 days. After 24 h of coculture in the presence of AD-CM, cancer cell conditioned medium or CA-CM (supplemented with 10% FBS), tumour cells were subjected to wound healing and Matrigel invasion assays.

### Cell viability assay

Breast cancer cells were seeded into a 96-well plate at 4000 cells per well in DMEM containing 10% FBS. After 12 h, the medium was replaced with serum-free, glucose-free DMEM, and the cells were cultured overnight. Then, the cells were treated with AD-CM, cancer cell conditioned medium or CA-CM for 24, 48, and 72 h. For the viability assay, methylthiazolyldiphenyl tetrazolium (MTT) (final concentration, 0.5 mol/l) was added to each well. The absorbance at 570 nm was measured using an ELISA reader (BioTek, Winooski, Vermont, USA) and used to determine the relative cell number in each well. The control cell viability was 100%.

### Measurements of metabolites in media

The β-hydroxybutyrate (Cayman), glycerol (Cayman), lactate (BioVision), pyruvate (BioVision), and FFA (BioVision) levels in media were measured using colorimetric assay kits according to the instructions from the manufacturer. The levels were normalized to protein concentration.

### Analysis of TG content

Tumour cells were grown with or without adipocytes for 3 days. Triglyceride (TG) content was quantified using a colorimetric kit (Cayman). The results were read at a wavelength of 570 nm by using an ELISA reader (BioTek, Winooski, Vermont, USA).

### Glucose uptake

Cells were seeded in 96-well black-bottom plates (4 × 10^4^ cells/well) and treated with glucose-free DMEM overnight. Then, the cells were cultured for 1 h with 2-nitrobenzodeoxyglucose (2-NBDG; final concentration, 100 μg/ml) in glucose-free DMEM with or without apigenin that reduced glucose uptake (Api; 50 μM) or insulin (INS; 50 μg/ml). The fluorescence was evaluated at 485/535 nm using a fluorescence plate reader (SpectraMax i3x, Molecular Devices, MD).

### Exosome isolation and characterization

After cells were cultured with exosome-depleted serum (Shin Chin Industrial, SCI), the exosomes were purified from the conditioned medium according to the instructions [16]. The medium was centrifuged at 500 *g* for five minutes and at 2000 *g* for thirty minutes at 4 °C to remove cellular debris and large apoptotic bodies. After centrifugation, media was added to an equal volume of a 2× polyethylene glycol (PEG, MW 6000, Sigma, 81,260) solution (final concentration, 8%). The samples were mixed thoroughly by inversion and incubated at 4 °C overnight. Before the tubes were tapped occasionally and drained for five minutes to remove excess PEG, the samples were further centrifuged at maximum speed (15,000 rpm) for 1 h at 4 °C. The resulting pellets were further purified using 5% PEG and then stored in 50–100 μl of particle-free PBS (pH 7.4) at − 80 °C. The average yield was approximately 300 μg of exosomal protein from 5 ml of supernatant. Total RNA was extracted by using Trizol reagent (Life Technologies), followed by miRNA assessment by microarrays and RT-PCR described below. Exosomes were analysed by electron microscopy to verify their presence, by a nanoparticle characterization system to measure their size and concentration, and by western blot to detect their proteins (HSP70, TSG101, CD63 and CD81).

### Electron microscopy

After being fixed with 2% paraformaldehyde, samples were adsorbed onto nickel formvar-carbon-coated electron microscopy grids (200 mesh), dried at room temperature, and stained with 0.4% (w/v) uranyl acetate on ice for 10 min. The grids were observed under a HITACHI HT7700 transmission electron microscope.

### Nanoparticle characterization system (NanoSight)

The NanoSight **(**Malvern Zetasizer Nano ZS-90) was used for real-time characterization and quantification of exosomes in PBS as specified by the manufacturer’s instructions.

### Exosome uptake analysis

Exosomes derived from breast cancer cells were labelled by the cell membrane labelling agent PKH26 (Sigma-Aldrich). After being seeded in 96-well plates and allowed to differentiate, mature 3T3-L1 cells were incubated with labelled exosomes (20 μl/well) for the indicated time. Images were acquired using the Olympus FluoView FV1000.

### Western blotting

After being washed twice with ice-cold PBS, cells were collected with SDS loading buffer and boiled for 10 min. The proteins were separated by SDS-PAGE, transferred to a nitrocellulose membrane, and detected with specific antibodies (Additional file 1: Table S2).

### RNA extraction and quantitative PCR

Gene expression was analysed using real-time PCR. The mRNA primer sequences are provided in Additional file 1: Table S3. The miRNA primer kits were purchased from RiboBio (Guang Zhou, China).

### Immunohistochemistry

A cohort of 106 paraffin-embedded human breast cancer specimens was diagnosed by histopathology at Renmin Hospital of Wuhan University from 2011 to 2012. Immunohistochemistry (IHC) staining was performed, and the staining results were scored by two independent pathologists based on the proportion of positively stained tumour cells and the staining intensity. The intensity of protein expression was scored as 0 (no staining), 1 (weak staining, light brown), 2 (moderate staining, brown) and 3 (strong staining, dark brown). The protein staining score was determined using the following formula: overall score = percentage score × intensity score. Receiver operating characteristic (ROC) analysis was used to determine the optimal cut-off values for all expression levels regarding the survival rate.

### miRNA microarrays

miRNA was isolated from exosomes with the miRNeasy Kit (Qiagen, USA), following the manufacturer’s instructions. miRNA levels were ascertained using TruSeq Small RNA Sample Prep Kits (Illumina, San Diego, CA, USA) according to the manufacturer’s instructions. ExomiRNA expression microarray data were deposited in the Gene Expression Omnibus (GEO) database (accession number: GSE109879).

### Luciferase assays

The 3′ UTRs of human target genes containing predicted miRNA binding sites (gene^wt^) were cloned into the GV272 vector (GeneChem Biotechnology, Shanghai, China), and the miRNA binding sites were replaced with a 4-nt fragment to produce a mutated 3′ UTR (gene^mut^) in the vector. Briefly, HEK 293 T cells were plated onto 12-well plates and grown to 70% confluence. The cells were cotransfected with gene^wt^ or gene^mut^, the pre-miRNA expression plasmid and pRL-SV40, which constitutively expresses Renilla luciferase as an internal control. Binding between TRAF6 and miRNA-146b was selected as the positive control [17]. At 48 h post-transfection, the cells were lysed, and Renilla luciferase activity was assessed by the TECAN Infiniti reader. The results are expressed as the ratio of firefly luciferase activity to Renilla luciferase activity.

### Extracellular acidification rate (ECAR) and oxygen consumption rate (OCR) analyses

Cells were seeded in 24-well XF24 cell culture plates at a density of 2 × 10^4^ cells/well for 24 h in CA-CM or AD-CM. Media were then removed, wells were washed, and the cells were incubated for 1 h at 37 °C without CO_2_ in XF modified DMEM assay medium (Seahorse Bioscience) at pH 7.4 supplemented with 1 mM glutamine, 2.5 mM glucose, 1 mM sodium pyruvate, 0.5 mM carnitine, and 1 mM palmitate complexed with 0.2 mM BSA. For glycolytic tests, the extracellular acidification rate (ECAR) was measured in the basal state (no glucose) or after the injection of 10 mM glucose, 5 μM oligomycin, and 50 mM 2DG (Sigma-Aldrich). For fatty acid oxidation (FAO) experiments, the oxygen consumption rate (OCR) was measured in the basal state (1 mM palmitate complexed with 0.2 mM BSA) or after the injection of 5 μM oligomycin, 1 μM FCCP (2-[2-[4-(trifluoromethoxy)phenyl] hydrazinylidene]-propanedinitrile), 5 μM rotenone and 5 μM antimycin A. ECAR is expressed as mpH per minute after normalization to protein content measured with a Pierce BCA Protein Assay (Thermo Fisher Scientific). OCR is expressed as pmol of O_2_ per minute after normalization to protein content.

### Lentivirus preparation and transfection

miRNA-144 and miRNA-126 inhibitors and pre-miRNA lentiviruses were obtained from GeneChem Biotechnology (Shanghai, China). Cells were cultured at 2 × 10^5^ cells/well in 6-well plates. After being incubated for 24 h, the cells were transfected with lentiviruses and control sequences using CON036 (GeneChem Biotechnology, China) following the manufacturer’s instructions. Cells (2 × 10^5^) were stably transfected with empty vector or with vectors carrying miRNA inhibitor or pre-miRNA using the TransIT-LT1 reagent (Mirus). Selection was carried out with puromycin (1 μg/ml, Sigma) or G418 (500 μg/ml, Sigma) in cell culture media for 48 h after transfection. Selected clones were maintained in DMEM with 500 μg/ml G418 or 1 μg/ml puromycin. Cell lysates were collected, and RT-PCR was performed to detect miRNA expression. The sequence information is provided in Additional file 1: Table S4.

### Xenograft tumour formation

Six-week-old female BALB/c nude mice were purchased from Vital River, Beijing. The animals were handled according to the protocol approved by the Institutional Animal Care and Use Committee of Renmin Hospital of Wuhan University. The following cell lines were used to create subcutaneous models: 2 × 10^6^ MDA-MB-231 cells treated with control lentivirus, transfected with miRNA-144 inhibitor lentivirus, or transfected with miRNA-126 inhibitor lentivirus. Breast cancer cells were injected alone or in combination with mature adipocytes (1 × 10^7^ cells). All cell samples were subcutaneously injected with Matrigel (1:1), total volume 100 μl, into the axilla of the mice. Tumour volume was defined as (longest diameter) × (shortest diameter)^2^/2 and was measured once every 4 days until day 32 using a Vernier calliper. For metastatic models, the abovementioned tumour cells (5 × 10^6^ cells) were injected alone through the tail vein. Lungs and livers were removed for assessment 30 days after tumour cell injection. After the mice were sacrificed, all tissues were collected, embedded in paraffin and stained with IHC or haematoxylin-eosin (HE).

### Statistical analysis

All experiments were done independently at least three times. The results are presented as the mean ± SD. The relative increase in protein expression was quantified using Image J software and was normalized to control protein expression in each experiment. Data sets obtained from different experimental conditions were compared with the t-test when comparing only 2 groups. Multiple comparisons between groups were performed using the Mann–Whitney *U* test or Tukey’s multiple comparisons. Survival probabilities for recurrence-free survival (RFS) were estimated using the Kaplan–Meier method, and variables were compared using the log-rank test. Pearson’s correlation was used to evaluate the correlations among monocarboxylate transporter 1 (MCT1), uncoupling protein 1 (UCP1) and MCT4 expression levels. In the bar graphs, a single asterisk (*) indicates *P* < 0.05.

### Data availability

The microarray data on exosomal miRNA expression in MDA-MB-231 cells cocultivated with mature 3T3-L1 cells were deposited in the GEO database with accession number GSE109879. The authors declare that all the other data supporting the findings of this study are available within the article and its Supplementary Information files and from the corresponding author upon reasonable request.

## Results

### Stromal adipocyte characteristics and metabolite biomarkers in breast cancer is linked to poor prognosis

Breast cancer cells invade regions of adipocytes in the tumour microenvironment [6]. Therefore, we assessed the possibility that stromal adipocytes contribute to the increased expression of beige/brown adipose biomarkers and catabolite transporters detected in samples from patients with breast cancer and determined the significance of these biomarkers for the overall survival of breast cancer. For these purposes, we initially detected the expression of UCP1, MCT1, MCT4, CD36 (also called fatty acid translocase), etc. in a cohort of 106 breast cancer specimens using immunohistochemistry (IHC). High expression of UCP1, a known marker of brown adipocytes [18], was detected specifically in resident adipose tissue (Fig. 1a). The presence of adipose tissue was also verified by perilipin A expression (Additional file 1: Figure S1). MCT1 and MCT4 are both catabolite transporters, MCT1 is an importer of monocarboxylates, such as lactate and pyruvate, while MCT4 primarily mediates the export of lactate and pyruvate [19]. In terms of fatty acid transport, CD36 binds long-chain fatty acids and facilitates their transport across the cell membrane, thus participating in lipid utilization and energy storage [20]. Fatty acid transport protein-1 (FATP1) enhances the intracellular accumulation of long chain fatty acids [21]. Regarding catabolite transporters, the expression of MCT1, CD36 and fatty acid transport protein-1 (FATP1) was detected in most breast cancer tissues with predominant localization proximal to adipose tissue, while the upregulated expression of MCT4 and CD36 and downregulated expression of fatty acid binding protein-4 (FABP4) were detected in most CAAs compared to normal mammary adipose tissue (Fig. 1a, Additional file 1: Figure S1). The previous study had indicated that high expression of UCP1 in stromal cells increases the production and the release of ketone body, which can be uptaken by cancer cells via overexpression of MCT4 [22]. Furthermore, our results showed that MCT4 expression was positively correlated with UCP1 expression in CAA specimens, and MCT1 expression in breast cancer tissue was positively correlated with MCT4 expression in local adipose tissue from breast cancer specimens (Fig. 1b).

**Fig. 1:** Elevated stromal adipocyte characteristics and metabolite biomarkers in breast cancer are linked to a poor prognosis. **a** Representative immunohistochemistry staining of UCP1, MCT4, MCT1, CD36, FABP4 and FATP1. The pictures show positive cytoplasmic staining for UCP1 and positive membrane staining for MCT4 and CD36 in stromal adipocytes from breast cancer specimens. The pictures also show positive staining for FATP1 and CD36 in breast cancer tissues located near stromal adipocytes. **b** Correlation analyses of protein expression levels among UCP1, MCT4, and MCT1. MCT4 versus UCP1 (up) and MCT1 (down). **c** Kaplan-Meier survival analysis of patients with biomarker-positive and biomarker-negative IHC staining, as well as analysis of the double-positive group versus the double-negative group

Kaplan-Meier analysis revealed that patients with MCT4 overexpression in adjacent adipose tissue had a poorer survival time than patients with MCT4 underexpression (Fig. 1c, P = 0.0115 and *P* = 0.005, log-rank test). Consistent results were obtained for the expression of FATP1 or CD36 in breast cancer tissue (Fig. 1c). However, UCP1 and MCT1 levels in the specimens were unrelated to poor survival. The correlation between MCT4 expression and poor prognosis in breast cancer was further strengthened when combined with high MCT1 *expression* (Fig. 1c). These findings suggest that high MCT4 expression in stromal adipose tissue and overexpression of CD36 or FATP1 in malignant tissue may serve as important clinical biomarkers for the poor prognosis of breast cancer patients.

### Cocultivated adipocytes exhibit increased beige/brown characteristics and supply metabolites to breast cancer cells

Adipocytes promote tumour growth and invasion in vitro and in vivo [5, 8, 23], but the mechanism by which they contribute to cancer metastasis remains controversial. Mature adipocytes cocultivated with breast cancer cells displayed a dramatic reduction in lipid droplet size, number and TG content (Fig. 2a). Moreover, our results demonstrated that tumour-surrounding adipocytes appeared to be undergoing a lipolytic process. Glycerol and FFAs, the products of TG hydrolysis, were released by adipocytes incubated with both MDA-MB-231 and MCF-7 cells (Fig. 2a). Similarly, pyruvate, lactate and the ketone body β-hydroxybutyrate accumulated in CAA conditioned medium (CA-CM) (Fig. 2b). To confirm if this change in adipocytes was indeed due to exosome uptake, we added cytochalasin D (CytoD), an endocytosis inhibitor, to mature 3T3-L1 culture media supplemented with exosomes purified from CA-CM. Notably, CytoD partially inhibited the increase in metabolites in CA-CM (Fig. 2b). As shown in Fig. 2c, glucose uptake was markedly reduced in adipocytes cultivated with CA-CM and stimulated with insulin, furthermore, the glucose uptake was accompanied by decreased expression of glucose transporter-4 (Glut-4) and insulin receptor substrate-1 (IRS1) (Fig. 2g). In parallel, the ECAR in response to glucose was increased in mature 3T3-L1 cells after coculture, demonstrating that anaerobic glycolysis was already maximal in cocultivated adipocytes in the presence of glucose. We then investigated the OCR in conditions that favour FAO (Krebs medium with palmitate, carnitine, and restricted glucose). In these conditions, the OCR was decreased in cocultivated cells compared with non-cocultivated cells (Fig. 2d). Likewise, increased matrix density in the ultrastructure of mitochondria, known to correlate with an increase in their activity, was also found in cocultivated adipocytes (Additional file 1: Figure S4). As tumour cells invade their surrounding environment, they induce the expression of the main rate-limiting enzymes in catabolic processes, such as glycolysis, TG hydrolysis and ketone body production in stromal tissues [5, 23, 24]. Adipocytes cocultivated with MDA-MB-231 cells showed enhanced levels of several rate-limiting enzymes, as exemplified by the robust increases in the mRNA levels of ATGL (adipose triglyceride lipase), LDH (lactate dehydrogenase A), BDH1 (3-hydroxybutyrate dehydrogenase 1), HMGCL (3-hydroxymethyl-3-methylglutaryl-CoA lyase) and HMGCS2 (3-hydroxy-3-methylglutaryl-CoA synthase 2), as well as in those of beige/brown markers such as PGC1-α and PRDM16, but the level of PDH (pyruvate dehydrogenase) was reduced (Fig. 2f, *P* < 0.05). Therefore, the results indicate that cocultivation-derived exosomes remodel metabolism in adipocytes.

**Fig. 2:** Adipocytes cocultivated with breast cancer cells present increased beige/brown adipocyte characteristics and undergo extensive metabolism changes. **a** Left, mature adipocytes in the presence or absence (NC) of MCF-7 or MDA-MB-231 tumour cells were stained with red oil. Right, the TG content in adipocytes. Breast cancer cells were transfected with miRNA-126 inhibitor, and then cocultured with mature adipocytes. The adipocytes in the CytoD group were treated with cytochalasin D (final concentration, 2 μg/ml) and 20 μg of exosomes purified from cancer-associated adipocyte conditioned medium (CA-CM). **b** The levels of secreted metabolites (glycerol, free fatty acids, pyruvate, lactate and β-hydroxybutyrate) enriched in media were determined by colorimetric assay. AD: adipocytes. **c** Glucose uptake was evaluated over time by 2-NBDG (50 μM) in glucose-free DMEM without or with insulin (INS) (50 μg/ml) or apigenin (Api) (50 μM), and the results are expressed as the mean fluorescence intensity (MFI). AD-126KD group: adipocytes cocultured with miR-126 knockdown breast cancer cells. **d** Raw data for the oxygen consumption rate (OCR) and extracellular acidification rate (ECAR) as determined by the Seahorse XF24 analyser. The ECAR was evaluated after the addition of 10 mM glucose to adipocytes in the presence or absence of breast cancer cells. The OCR was measured in the presence of palmitate as described in the Methods. **e** 3T3-L1 cells were marked with LC3II-positive autophagy membranes. Autophagy membranes (LC3) visible in the GFP and RFP channels after coculture with or without MDA-MB-231 cells are shown. Green fluorescence showed that LC3-I distributed in cytoplasm. Red fluorescence showed that LC3-II distributed in autophagolysosomes. Arrowheads show LC3-II-RFP(+) only autophagosomes. **f** Adipocytes were cocultivated in the presence or absence of breast cancer cells. After 3 days, mRNA was extracted for qPCR analysis of the expression of the indicated genes, and (**g**) proteins were extracted for western blot analysis of the expression of the indicated proteins. Data are presented as the mean ± S.D. of at least three independent experiments. * *P* < 0.05 versus control values as blank group, # *P* < 0.05 versus control values as positive group

Previous studies have shown that mammary fat in the tumour microenvironment overexpresses UCP1 and exhibits a catabolic stroma [25]. Thus, we next evaluated if adipocytes undergo beige/brown differentiation, as assessed by the upregulation of UCP1 and the induction of a catabolic stromal phenotype. First, we assessed the levels of UCP1, MCT4 and CAV-1, which are hallmarks of metabolic stress associated with poor survival in breast cancer [26, 27]. Figure 2g shows that adipocytes cocultivated with tumour cells harboured increased UCP1 and MCT4 levels and induced Cav-1 loss compared with adipocytes cultivated alone. We next found elevated CD36 expression but significantly lower FABP4 expression in adipocytes cocultivated with breast cancer cells than in adipocytes alone (Fig. 2g); these results were similar to those reported in a previous study [28, 29]. We next evaluated the expression levels of p-AMPK, PPARγ, HIF1-α and LC3I/II as primary markers of catabolic modulation. Figure 2g shows that p-AMPK and HIF-1α were upregulated and that autophagy was induced, as evidenced by the upregulation of LC3II, in adipocytes incubated with both MDA-MB-231 and MCF-7 cells relative to normal adipocytes. Autophagic flux was also evident in 3T3-L1 cells expressing GFP-cherry-LC3 (Fig. 2e); few yellow dots were observed under control conditions, and green fluorescence showed a mostly uniform cytoplasmic distribution. Red dots were primarily observed in these cells, indicative of autophagolysosomes under conditions of basal autophagy. The protein level of PPARγ, which is involved in lipid accumulation, was dramatically reduced in cocultivated adipocytes (Fig. 2g). This finding was supported by the use of propranolol, the PPARγ activator, which partially reverses cancer cell–induced lipolytic activation [23]. Taken together, the findings indicate that cancer cells induce the beige/brown differentiation of adipocytes and promote adipocyte catabolism.

### Tumour cells cocultivated with mature adipocytes exhibit an aggressive phenotype

As demonstrated in a previous study, mature adipocytes stimulate the invasive ability of breast cancer cells by inducing incomplete EMT [5, 6]. Thus, we questioned whether adipocytes mimic the effects induced by coculture. As shown in Fig. 3a, the viability of breast cancer cells dramatically increased after exposure to CA-CM compared with control treatment. Moreover, the migration abilities of both MDA-MB-231 and MCF-7 cells in a wound healing assay were significantly increased with CA-CM compared with controls at 24 h (Fig. 3b). An invasion assay also demonstrated a profound increase in the number of invasive cells in the presence of CA-CM (Fig. 3c). Human breast cancer cells were cultivated in Transwells for 3 days in the absence or presence of mature murine adipocytes. The downregulation of E-cadherin, an EMT-related marker, was observed in the presence of mature 3T3-L1 cells relative to the absence of mature adipocytes (Fig. 3d). Hence, our results show that adipocytes promote breast tumour cell invasiveness in vitro.

**Fig. 3:** Tumour cells exhibit increased growth and invasion capacities upon coculture with adipocytes. Cancer-associated adipocyte conditioned medium (CA-CM) was collected from adipocytes cultivated with MCF-7 or MDA-MB-231 cells for 3 days, and adipocyte-conditioned medium (AD-CM) and cancer cell-conditioned medium were collected from cells cultivated alone under similar conditions for 3 days as controls. All media contained 10% FBS. **a** Cell viability was measured by MTT assay at 24, 48 and 72 h. **b** Wound healing assays were used to examine the effects of CA-CM on cell motility. The migration rate correlates with cell migration ability. **c** Tumour cells were cultivated in cancer cell-conditioned medium, AD-CM, or CA-CM. After 24 h, the number of cells penetrating the membrane in Transwell invasion assays was analysed. **d** E-cadherin protein expression was analysed by western blot in extracts from tumour cells cocultivated in the presence or absence of adipocytes (3 days). The bars represent the mean ± SD of triplicate datapoints (*n* = 3). * *P* < 0.05 versus control values

### Mature adipocytes alter breast cancer cell metabolism

First, we investigated whether coculture with adipocytes leads to alterations in the metabolism of breast cancer cells, as previously shown [23, 30]. Cocultivated MDA-MB-231 and MCF-7 cells exhibited multiple small lipid droplets as revealed by red oil (Fig. 4a). The TG concentration clearly increased in cocultivated cells, in accordance with lipid droplet accumulation (Fig. 4a). Likewise, glucose uptake was markedly increased in tumour cells cocultivated with adipocytes and was further increased after insulin stimulus (Fig. 4b). Surprisingly, we observed that cocultivated cells increased ECAR and decreased OCR in the presence of compared to non-cocultivated cells. This suggest that the increased FAO in cocultivated cells was not coupled to ATP production (Fig. 4c). Subsequently, the overexpression of MCT1, CD36 and FATP1 protein and FABP5 mRNA (Fig. 4d-e) in breast cancer cells in the presence of adipocytes indicated that tumour cells absorb more monocarboxylic acids (MAs, refer to pyruvate and lactate) and FFAs. Since we demonstrated that the tumour-surrounding adipocytes underwent glycolytic and lipolytic processes, it can be suggested that the lipids accumulating in the tumour cells originated from adipocytes. Our results show that the MAs and lipid transfer between adipocytes and tumour cells lead to TG storage in breast tumour cells and enhance glucose uptake by breast cancer cells.

**Fig. 4:** Breast cancer cells undergo metabolic adaptation in the presence of adipocytes. **a** Left, tumour cells cocultivated with or without mature adipocytes were stained with red oil. Right, the TG content in tumour cells. **b** Glucose uptake was evaluated over time by 2-NBDG (50 μM) in glucose-free DMEM without and with insulin (INS) (50 μg/ml) or apigenin (Api) (50 μM), and the results are expressed as the mean fluorescence intensity (MFI). AD: adipocytes. **c** Raw data for the OCR and ECAR as determined by the Seahorse XF24 analyser. The ECAR was evaluated after the addition of 10 mM glucose to tumour cells in the presence or absence of adipocytes. The OCR was measured in the presence of palmitate as described in the Methods. **d** MDA-MB-231 cells were cocultivated in the presence or absence of adipocytes. After 3 days, protein was extracted for western blot analysis of the expression of the indicated proteins, and (**e**) mRNA was extracted for the qPCR analysis of the expression of the indicated genes. Data are presented as the mean ± S.D. of at least three independent experiments. * *P* < 0.05 versus control values

Furthermore, we investigated whether adipocyte-derived FFAs are used for FAO. When tumour cells were cocultivated with adipocytes, AMPK was activated, as evidenced by phosphorylation of the conserved Thr172 residue in the catalytic subunit (Fig. 4d). Mitochondrial biogenesis, which facilitates the oxidative catabolism of both FFAs and glucose, is a vital process activated by AMPK. Additionally, AMPK phosphorylates and inactivates acetyl-CoA carboxylase (ACC) to promote FFA uptake into mitochondria. As shown in Fig. 4d, ACC phosphorylation was 3.4- and 1.7-fold increased respectively in cocultivated cells, and CPT1α, which transports fatty acyl chains from the cytosol into mitochondria to produce ATP from FAO, was also overexpressed in breast cancer cells exposed to adipocytes compared with those cultured alone. Similar results were previously observed in other studies [24, 30]. Additionally, the protein level of fatty acid synthase (FASN) was markedly decreased in breast cancer cells incubated with adipocytes, and FASN is modulated by AMPK-mediated phosphorylation and P38-regulated degradation [31, 32]. Simultaneously, p-P38 levels activated by p-AMPK were notably increased, providing further verification of FASN modulation. In addition, acetyl-CoA acetyltransferase 1/2 (ACAT1/2) and 3-oxoacid CoA-transferase 1/2 (OXCT 1/2), enzymes associated with ketone re-utilization, were increased at the mRNA level in breast cancer cells in the presence of adipocytes (Fig. 4e), indicating that breast cancer cells allow ketone body re-utilization to maintain tumour growth. Therefore, cocultivated cancer cells increase MAs and FFA uptake by increasing their transporters, and AMPK is activated to inhibit lipid biosynthesis and promote uncoupled FAO through the ACC/CPT1α axis and FASN downregulation, leading to a persistent state of metabolic remodelling.

### Cocultivated breast cancer cells show altered exosomal miRNA profiles

Exosomes were isolated from conditioned medium derived from MDA-MB-231 cells cocultivated with mature adipocytes for 3 days. The purified particles displayed typical exosome morphology and size and contained CD63, TSG101 and CD81 but not HSP70 (Fig. 5a-c), which was consistent with previous reports on exosomes [10]. To observe exosome uptake by adipocytes, breast cancer-secreted exosomes were labelled with red fluorescence. After being treated with tumour exosomes for 4 h, mature 3T3-L1 cells were densely packed with exosomes (Fig. 5d), indicating rapid cellular uptake of exosomes by adipocytes.

**Fig. 5:** Breast cancer cells cocultured with adipocytes show altered exosomal miRNA expression profiles. **a** Exosomes originating from CA-CM viewed by electron microscopy (scale bar, 200 nm). **b** Exosomes from CA-CM were analysed by western blot. **c** NanoSight analysis of exosomes derived from MDA-MB-231 cells and CA-CM. **d** Labelled tumour cell-secreted exosomes (red) were incubated with the indicated adipocytes. The adipocytes were treated with and 20 μg of exosomes purified from cancer medium (CM). **e** miRNA microarray analysis of purified exosomes from MDA-MB-231 cells and CA-CM. The heatmap shows the top 20 differentially expressed miRNAs between the two groups. **f** MDA-MB-231 or MCF-7 cells were cocultivated in the presence or absence of adipocytes. After 3 days, exosomal miRNAs were further verified by qPCR. **g** Adipocytes were cocultivated in the presence or absence of tumour cells. After 3 days, RNA was extracted from the adipocytes and subjected to qPCR analysis with primers specific to mature miRNA. Data are presented as the mean ± S.D. of at least three independent experiments. * *P* < 0.05 versus control values

Many studies have confirmed that miRNAs can be transported between tumour cells and stromal cells, such as fibroblasts, macrophages and endothelial cells [33]. Therefore, we attempted to identify the miRNA content that was transferred from breast cancer cells to adipocytes. miRNA microarrays were utilized to analyse exosomes in CA-CM, and exosomes from MDA-MB-231 cells alone were extracted from a GEO dataset (GSE50429) as a control. The exosomal miRNA sequencing analysis revealed distinct differences between the exo-miRNA profiles derived from normal MDA-MB-231 cells and CA-CM. The top 20 differentially expressed miRNAs in exosomes from CA-CM are shown in Fig. 5e. To confirm the sequencing results, qRT-PCR was performed to investigate the expression of 10 exomiRNAs in media from adipocytes, MCF-7 cells and CA-CM/MCF-7 cells. There were differences in exomiRNA expression between incubated MDA-MB-231 and MCF-7 cells; miRNA-21 and miRNA-22 expression levels were decreased in CA-CM/MCF-7 cells but were increased in CA-CM/MDA-MB-231 cells based on the microarray analysis (Additional file 1: Figure S2A). miRNAs are encapsulated in exosomes in a selective or concentration-dependent manner, and thus, these miRNA expression profiles in the cells were analysed using UCSC (https://xenabrowser.net/heatmap) (Additional file 1: Figure S2B). Ultimately, we selected miRNA-144 and miRNA-126 for further investigation. Among the most highly expressed miRNAs in the exosome microRNA profile, miRNA-144 and miRNA-126 showed much higher expression levels in CA-CM exosomes than in control exosomes, and this finding was confirmed by RT-PCR (Fig. 5e-f). In addition, the treatment of MDA-MB-231 cells with GW4869, which is reported to inhibit the secretion of exosomes from cells [34], resulted in a reduction in miRNA-126 secretion in CA-CM exosomes (Additional file 1: Figure S2C). The expression of mature miRNA-144 and mature miRNA-126 was significantly increased in adipocytes cultivated with MDA-MB-231 cells compared to adipocytes cultured alone, while the pre-miRNA levels were not detected in either group (Fig. 5g). By contrast, mature miRNA-155 expression was upregulated in adipocytes cultivated with tumour cells, while there was no disparity in pre-miRNA-155 levels between cocultured adipocytes and those cultivated alone (Additional file 1: Figure S2D). Together, these data support that breast cancer cells cocultivated with adipocytes show increased expression of miRNA-144 and miRNA-126 expression, which are subsequently released via the exosome pathway.

### Exosomal miRNA-144 from breast cancer cells mediates the beige/brown adipocyte characteristic

To determine the mechanism by which exosomal miRNA-144 dysregulation leads to the beige/brown differentiation of adipocytes, we attempted to identify target genes and pathways modulated by miRNA-144. Previous studies demonstrated that miRNA-144, acting as a negative regulator, directly binds to the 3′-UTR of MAP3K8 and inhibits ERK1/2 phosphorylation [35]; thus, MAP3K8 was assumed to be a particularly relevant miRNA-144 target gene.

One potential conserved seed site was identified by TargetScan, PicTar and miRBase upon alignment of miRNA-144 with the human MAP3K8 3’UTR sequence (Fig. 6a). We next established a luciferase reporter containing the human MAP3K8 3’UTR and cotransfected it with pre-miRNA-144 mimic or pre-miRNA-control into HEK 293 cells. We also used a MAP3K8 3’UTR construct harbouring a mutation in the predicted miRNA-144 site as a control. The results showed a significant decrease in normalized luciferase activity of the wild-type construct in the presence of human pre-miRNA-144 relative to control, while this luciferase activity was rescued by the mutated 3’UTR of human MAP3K8 (Fig. 6b). This finding suggests that MAP3K8 is indeed a direct target of miRNA-144.

**Fig. 6:** miRNA-144 suppresses the beige/brown differentiation of adipocytes by downregulating MAP3K8, and miRNA-126 remodels adipocyte metabolism by downregulating IRS-1. The adipocytes in the cytochalasin D (CytoD) group were treated with CytoD (final concentration, 2 μg/ml) and 20 μg of exosomes purified from cancer-associated adipocyte conditioned medium (CA-CM). **a** The predicted miRNA-144 binding site in the 3’UTR of the MAP3K8 gene and the predicted miRNA-126 binding site in the 3’UTR of the IRS-1 gene from TargetScan. **b** The GV272 vector containing the 3’UTR of the target gene harbouring wild-type (wt) or mutated (mt) miRNA binding sites was transfected into HEK 293 T cells stably expressing miRNA or empty vector (as a control). Luciferase activity was analysed at 48 h post-transfection, and the ratio of firefly luciferase activity to Renilla luciferase activity is shown. **c** Breast cancer cells were transfected with miRNA-126 inhibitor, mature adipocytes were transfected with miRNA-126 mimic as the positive control and the control vector was applied as the negative control. Mature adipocytes cultured in the presence or absence of tumour cells for 3 days were stained with red oil (**d**), and mRNAs were extracted for the qPCR analysis of the expression of the indicated genes. **e**, **f** Western blot analysis of related protein expression in different groups. Data are presented as the mean ± S.D. of at least three independent experiments. * *P* < 0.05 versus control values

As MAP3K8 downregulates ERK1/2 phosphorylation, we investigated whether the decreased ERK1/2 phosphorylation levels in cocultured adipocytes are associated with an increase in exomiRNA-144 expression. We transfected pre-miRNA-144 into mature 3T3-L1 cells as the positive control group and treated mature 3T3-L1 cells with exosomes from CA-CM and CytoD. We observed that ERK1/2 phosphorylation levels significantly decreased in adipocytes incubated with breast cancer cells and adipocytes overexpressing miRNA-144, while both miRNA-144 knockdown in cultured breast cancer cells and CytoD treatment rescued the reduced ERK1/2 phosphorylation levels in adipocytes cultured with breast cancer cells (Fig. 6e). A previous study has shown that ERK1/2 phosphorylates PPARγ at S273, and the inhibition of PPARγ phosphorylation at S273 induces UCP1 overexpression in adipocytes [36]. Similarly, we showed that the levels of both total and phosphorylated (S273) PPARγ were notably reduced in adipocytes incubated with breast cancer cells and in adipocytes overexpressing miRNA-144, whereas these levels were restored upon miRNA-144 knockdown in cultivated breast cancer cells and upon treatment with CytoD (Fig. 6e). These consistent results were confirmed by UCP1 expression (Fig. 6e). Altogether, these experiments demonstrate that miRNA-144, which is derived from cultivated exosomes, mediates the beige/brown differentiation of adipocytes thorough the downregulation of the MAP3K8/ERK1/2/PPARγ axis.

### Exosomal miRNA-126 from breast cancer cells mediates adipocyte metabolism remodelling

Previous studies have reported that IRS1 is the functional downstream target of miRNA-126 via its 3’UTR [37], and the alignment of miRNA-126 with the human IRS1 3’UTR sequence revealed one potential conserved seed site (Fig. 6a). The luciferase activity in the IRS1^wt^ group induced by human pre-miRNA-126 was dramatically decreased compared to that in the control group, while this activity was restored using the mutated 3’UTR of human IRS1 (Fig. 6b). These data demonstrate that IRS1 is indeed a direct target of miRNA-126.

To understand if miRNA-126 can modulate adipocyte metabolism by targeting IRS1, we investigated that whether exosomal miRNA-126 alters glucose and lipid homeostasis in adipocytes. By contrast, mature adipocytes in the presence of breast cancer cells and miRNA-126 inhibition regained lipid droplet accumulation compared to the positive control (Fig. 6c). Similar results were observed regarding the levels of key enzymes involved in lipid metabolism (Fig. 6d). As shown in Fig. 6f, IRS1 was suppressed in adipocytes cocultivated with tumour cells and in adipocytes overexpressing ectopic miRNA-126, while silencing miRNA-126 in cultivated breast cancer cells or treating cells with CytoD restored IRS1 expression. Moreover, decreased Glut-4 expression was observed in adipocytes cultured with breast cancer cells, while Glut-4 levels were high in miRNA-126-overexpressing adipocytes (Fig. 6f), which showed reduced glucose uptake [38]. Previous work has demonstrated that miRNA-126 activates and stabilizes hypoxia-inducible factor-1α (HIF-1α), which activates the expression of both pyruvate dehydrogenase kinase 1 (PDK1) and lactic dehydrogenase A (LDHA) to switch cells from oxidative to glycolytic metabolism [39]. To assess whether exomiRNA-126 induces HIF-1α expression, HIF-1α protein levels were shown to be upregulated in adipocytes incubated with breast cancer cells and in miRNA-126-transfected adipocytes (Fig. 6f). Here, adipocytes cocultured with breast cancer cells or transfected with miRNA-126 mimic induced AMPK phosphorylation, which in turn triggered autophagy, as assessed by the accumulation of LC3II (Fig. 6f). In summary, our results indicate that exomiRNA-126 induces complex metabolic remodelling in adipocytes, including catabolic induction following the disruption of IRS/Glut-4 signalling, the activation of the AMPK/autophagy pathway, and the stabilization of HIF1α expression.

### Blockade of miRNA-144 or miRNA-126 reduces adipocyte-induced tumour growth in vivo

To study the in vivo effect of exosomal miRNA-144 or miRNA-126 intervention, we monitored the in vivo tumour growth of miRNA-144-knockdown or miRNA-126-knockdown MDA-MB-231 cells co-injected with mature 3T3-L1 cells or control cells in the mammary and axilla fat pads of mice. Mice in the normal control group were injected with MDA-MB-231 cells and PBS, while those in the positive control group were injected with MDA-MB-231 cells cocultivated with mature adipocytes. We measured tumour volume every 4 days for 32 days, and found that significantly increased tumour growth in mice co-injected with MDA-MB-231 cells and mature 3T3-L1 cells compared with those in the normal control group (Fig. 7a). In addition, the mice in the miRNA-144- or miRNA-126-knockdown groups developed smaller tumours than those in the positive control group (Fig. 7b). Likewise, the number and the size of metastatic nodules in the lungs and liver were markedly increased in the group injected with tumour cells cocultivated with mature 3T3-L1 cells relative to the control group, while the tumours were significant smaller in the mice injected with miRNA-126-inhibited or miRNA-144-inhibited tumour cells (Fig. 7c-d). Meanwhile, the number of Ki67-positive cells determined using IHC staining and the nuclear grade assessed by HE staining, which indicates the rate of cell proliferation, were prominently increased in mice co-injected with MDA-MB-231 cells and mature 3T3-L1 cells, while these values were decreased in mice injected with miRNA-126- or miRNA-144-knockdown cells (Fig. 7d). Thus, these data confirm that higher exomiRNA-144 and exomiRNA-126 expression in the microenvironment plays an important role in breast cancer progression.

**Fig. 7:** Blockade of miRNA-144 or miRNA-126 reduces adipocyte-induced tumour growth in vivo. **a** miRNA-144-knockdown MDA-MB-231 cells or miRNA-126-knockdown MDA-MB-231 cells were co-injected with mature 3T3-L1 cells into the mammary and axilla fat pads of mice. As a control, normal MDA-MB-231 cells mixed with or without adipocytes in Matrigel were inoculated into the mammary and axilla fat pads of ten BALB/c nude mice (9 mice in each group). Tumour size was measured every 4 days starting at day 32. **b** Representative tumour images from nine mice. **c** Macrometastatic lesions were observed in the liver or lungs (arrows). **d** Proliferating cells in tumours were detected by IHC staining using an anti-Ki67 antibody, and HE staining was performed for the histologic analysis of tumours, lungs and liver. Scale bar, 100 μm. Data are presented as the mean ± S.D. of at least three independent experiments. * *P* < 0.05 versus control values

## Discussion

While crosstalk between adipocytes and cancer cells has been described in previous studies [5, 8, 23]. Previous studies have shown interaction entails a vicious circle, wherein breast cancer cells transform adipocytes, which, in turn, promote tumour progression. Soluble factors, such as inflammatory factors and adrenomedullin, have been demonstrated to be involved in this process [6, 40]. However, the role of exosomes was previously unknown.

Here, we show an important role for exosomes originated from the tumour-adipocytes interaction in a complex metabolic network favouring malignant progression that is established between breast cancer cells and adipocytes at the tumour invasive front.

The preliminary step of this symbiosis is the ability of tumour cells to induce beige/brown differentiation and the lipolytic process in adipocytes. Our results showed that adipocytes presented beige/brown characteristics and an activated phenotype, assessed by the induction of autophagy and the overexpression of catabolic enzymes and efflux transporters in the breast cancer microenvironment. As shown in previous studies, cancer-associated fibroblasts (CAFs) overexpress UCP1 to significantly promote breast cancer growth via the production of high-energy mitochondrial fuels containing lactate, pyruvate and FFAs [26]. Furthermoremultiple key enzymes in the catabolic process are increased in tumour-surrounding adipocytes, which is consistent with our results [30]. Moreover, beige/brown adipose markers are enriched in host cells to stimulate tumour growth [41], and autophagy is activated by upregulating UCP1 levels, inducing lipolysis and generating metabolites [26, 42]. In addition, AMPK, which was observed to be highly activated in stromal adipocytes in our study, phosphorylates ATGL at S406 and HSL at S565 to stimulate lipolysis [43], acutely regulates glycolysis by phosphorylating PFKFB3 (6-phosphofructo-2-kinase/fructose-2,6-biphosphatase 3) [44], and induces ketogenesis through the activation of PPARα [45]. Thus, these data demonstrate that upon crosstalk with breast cancer cells, adipocytes increase catabolism and transfer energy to sustain tumour cell invasion.

Tumour cells adjoining stromal adipocytes have previously been shown to exert significant changes in proliferation, migration, and invasion. The ability of adipocytes to modify tumour progression has been reported in ovarian cancer [23], melanoma [46] and pancreatic cancer [47]. Several observations have also shown that breast cancer cells cocultivated with mature adipocytes exhibit an enhanced invasive phenotype by decreasing E-cadherin expression and increasing the expression of mesenchymal markers [5]. Similarly we showed that breast cancer cells cocultivated with adipocytes enhanced their invasive capacity by reducing E-cadherin levels. In addition, breast cancer cells in an adipocyte-rich microenvironment have increased UCP2 expression, which leads to uncoupled FAO and reduced ATP generation, further activating AMPK [30]. Similarly, our results demonstrated that adipocyte-released metabolic intermediates are transferred to breast cancer cells, which increased fatty acid uptake by overexpressing CD36 and FATP1 and accelerated FAO through the AMPK/ACC2/CPT1α axis, as previously reported [43, 48]. In contrast, breast cancer cells increasingly took in lactate, pyruvate and ketone bodies to supply energy by increasing MCT1 levels. Intriguingly, breast cancer cells strongly overexpressed levels of ATGL, BDH1, HMGCL and HMGCS2, but decreased the level of PDH. This suggests that breast cancer cells mainly depended on the energy supply via oxidation of fatty acids and ketones instead of pyruvate and is consistent with other research [49]. Taken together, the data indicate that breast cancer cells, acting as metabolic parasites, constantly seized energy and biomass from local adipocytes to fuel tumour growth and metastasis.

Exosomes play a pivotal role in the metabolic symbiosis between adipocytes and multiple types of cancer cell [46]. Recent results indicate that exosomes derived from adipocytes carry proteins that promote cancer cell migration and invasion by increasing FAO [46]. While exosomes secreted by pancreatic cancer cells induce lipolysis in subcutaneous adipose tissue [40] these studies suggest that exosomes have bidirectional effects on the interactions between cancer cells and adipocytes. Our study revealed the exomiRNA-144, acting as an important communicator between tumour cells and adipocytes, promoted the beige/brown differentiation of adipocytes, and exomiRNA-126 also played a vital role in the metabolic reprogramming of adipocytes. miRNA-144 serves as a tumour suppressor in multiple cancers [35]. However, breast cancer cells, such as SKBR3 and MDA-MB-231 cells, exhibit dramatically increased radiation resistance after miRNA-144 overexpression [50]. Moreover, Vivacqua and colleagues reported that 17β-estradiol triggered the induction of miRNA-144 in CAFs, which are the main components of the tumour microenvironment driving cancer progression [51]. Thus, it appears that miRNA-144 might be regarded as a stress-associated inducer.

By contrast, miRNA-126 is regarded as a metastasis suppressor in breast cancer [52], and exomiRNA-126 originates from tumour-induced blood vessel formation and malignant transformation [53]. In addition, miRNA-126 is upregulated and secreted by exosomes under conditions of oxidative stress and hypoxia [37], indicating that exomiRNA-126 from cancer cells might be involved in tumour angiogenesis. Tomasetti and colleagues reported that miRNA-126 targets IRS1 and further stabilizes HIF-1α by inducing citrate accumulation in the cytoplasm and activates autophagy by remodelling cell metabolism [37, 38], suggesting its involvement in the metabolic dysfunction of stromal adipocytes. Surprisingly, decreased Glut-4 levels and glucose uptake are observed in cocultivated adipocytes overexpressing HIF-1α, which promotes Glut-4 expression [39]. There is evidence that PPARγ loss attenuates the activation of hypoxia-responsive genes while increasing the levels of inflammatory genes, such as CCL5, in mature hypoxic adipocytes [54]. PPARγ levels were confirmed to decrease in our study, while CCL5 levels in the medium increased (Additional file 1: Figure S3). Moreover, exomiRNA-122 was highly expressed but was not extensively studied, and exomiRNA-122 inhibits glucose uptake in premetastatic niche cells by downregulating the glycolytic enzyme pyruvate kinase to facilitate disease progression [55]. Likewise, the expression of miRNA-155, which causes an increased inflammatory state in adipocytes via its ability to target PPARγ mRNA [56], was also upregulated in our study. Taken together, the results show that exomiRNAs are probably exploited by cancer cells as a sort of ‘signal’ to convert the cells in the microenvironment into a pro-tumour niche.

## Conclusions

In conclusion, we discovered that exosomes containing miRNA-144 and miRNA-126 are highly secreted from breast cancer cells co-cultured with adipocytes and promote metastasis by inducing beige/brown differentiation and reprogramming the metabolism in surrounding adipocytes. Our work suggests a new mechanism for the interaction between stromal cells and cancer cells mediated by exomiRNAs, and the development of therapeutics to block this interaction will be a promising strategy in cancer therapy.

## Additional file

Additional file 1: **Figure S1.** The expression of Perilipin A and FAPB4 in invasive front of breast cancer. **Figure S2.** miRNA expression in exosomes and tumor cells. **Figure S3.** The level of CCL5 in the supernatants of adipocytes increased in the presence of breast tumor cells. **Figure S4.** Representative experiments of transmission electron microscopy highlighting mitochondrial ultra-structural changes (*) in adipocytes or adipocytes cultivated with MDA-MB-231. **Table S1.** Patient characteristics. **Table S2.** Antibody information. **Table S3.** The primers sequences of mRNA and the primers sequences of miRNA purchased from (RIBBIO, Guangzhou China). **Table S4.** The sequences of plasmids and lentiviruses. (PPTX 3373 kb)

## Abbreviations

ACAT: Acetyl-CoA acetyltransferase
ACC: Acetyl-CoA carboxylase
ACLY: Citrate lyase
AD-CM: Adipocytes conditioned medium
Api: Apigenin
ATGL: Adipose triglyceride lipase
BDH1: 3-hydroxybutyrate dehydrogenase 1
CAAs: Cancer-associated adipocytes
CA-CM: Cancer-associated adipocytes conditioned medium
CAFs: Cancer-associated fibroblasts
CPT1: Carnitine palmitoyltransferase I
CytoD: Cytochalasin D
EMT: Epithelial-mesenchymal transition
FABP: Fatty acid binding protein
FAO: Fatty acid oxidation
FASN: Fatty acid synthase
FATP: Fatty acid transport protein
FBS: Fetal bovine serum
FCS: Fetal calf serum
FFAs: Free fatty acids
GEO: Gene Expression Omnibus
Glut-4: Glucose transporter-4
HE: Hematoxylin-Eosin
HIF-1α: Hypoxia inducible factor 1 α
HMGCL: 3-hydroxymethyl-3-methylglutaryl-CoA lyase
HMGCS2: 3-hydroxy-3-methylglutaryl-CoA synthase 2
HRs: Hazard ratios
HSL: Hormone-sensitive lipase
IGF1: Insulin-like growth factor-1
IHC: Immunohistochemistry
IRS1: Insulin receptor substrate-1
KM: Kaplan-Meier
LDHA: Lactate dehydrogenase A
MAs: Monocarboxylic acids
MCT: Monocarboxylate transporter
OS: Overall survival
OXCT: 3-oxoacid CoA-transferase
PDH: Pyruvate dehydrogenase
PDK1: Pyruvate dehydrogenase kinase 1
PFKFB3: 6-phosphofructo-2-kinase/fructose- 2,6-bisphosphatase 3
PGC1-α: PPARγ coactivator-1α
PPARγ: Peroxisome proliferators activated receptor γ
PRDM16: PR domain containing 16
RFS: Recurrence-free survival
SFA: Saturated fatty acid
TG: Triglyceride
UCP1: Uncoupling protein 1
